The article "Genome-wide identification and characterization of TALE superfamily genes in cotton reveals their functions in regulating secondary cell wall biosynthesis" was retracted in 2024. Reasons: duplicated images; original data or images not available; unreliable results or conclusions; concerns about the data.

# Genome-wide identification and characterization of TALE superfamily genes in cotton reveals their functions in regulating secondary cell wall biosynthesis

**DOI:** 10.1186/s12870-019-2026-1

**Published:** 2019-10-17

**Authors:** Qiang Ma, Nuohan Wang, Pengbo Hao, Huiru Sun, Congcong Wang, Liang Ma, Hantao Wang, Xianlong Zhang, Hengling Wei, Shuxun Yu

**Affiliations:** 1 State Key Laboratory of Cotton Biology, Institute of Cotton Research, Chinese Academy of Agricultural Sciences, Key Laboratory of Cotton Genetic Improvement, Ministry of Agriculture, Anyang, 455000 Henan China; 2 College of Plant Science & Technology, Huazhong Agricultural University, Wuhan, 430070 Hubei China

**Keywords:** *Gossypium* spp., Genome-wide, TALE transcription factors, Secondary cell wall, QTLs colocalization, Protein interaction, Regulatory network

## Abstract

**Background:**

Cotton fiber length and strength are both key traits of fiber quality, and fiber strength (FS) is tightly correlated with secondary cell wall (SCW) biosynthesis. The three-amino-acid-loop-extension (TALE) superclass homeoproteins are involved in regulating diverse biological processes in plants, and some TALE members has been identified to play a key role in regulating SCW formation. However, little is known about the functions of TALE members in cotton (*Gossypium* spp.).

**Results:**

In the present study, based on gene homology, 46, 47, 88 and 94 TALE superfamily genes were identified in *G. arboreum*, *G. raimondii*, *G. barbadense* and *G. hirsutum,* respectively. Phylogenetic and evolutionary analysis showed the evolutionary conservation of two cotton TALE families (including BEL1-like and KNOX families). Gene structure analysis also indicated the conservation of GhTALE members under selection. The analysis of promoter cis-elements and expression patterns suggested potential transcriptional regulation functions in fiber SCW biosynthesis and responses to some phytohormones for GhTALE proteins. Genome-wide analysis of colocalization of TALE transcription factors with SCW-related QTLs revealed that some BEL1-like genes and KNAT7 homologs may participate in the regulation of cotton fiber strength formation. Overexpression of *GhKNAT7-A03* and *GhBLH6-A13* significantly inhibited the synthesis of lignocellulose in interfascicular fibers of *Arabidopsis*. Yeast two-hybrid (Y2H) experiments showed extensive heteromeric interactions between GhKNAT7 homologs and some GhBEL1-like proteins. Yeast one-hybrid (Y1H) experiments identified the upstream GhMYB46 binding sites in the promoter region of GhTALE members and defined the downstream genes that can be directly bound and regulated by GhTALE heterodimers.

The article "Genome-wide identification and characterization of TALE superfamily genes in cotton reveals their functions in regulating secondary cell wall biosynthesis" was retracted in 2024. Reasons: duplicated images; original data or images not available; unreliable results or conclusions; concerns about the data.

**Conclusion:**

We comprehensively identified TALE superfamily genes in cotton. Some GhTALE members are predominantly expressed during the cotton fiber SCW thicking stage, and may genetically correlated with the formation of FS. Class II KNOX member GhKNAT7 can interact with some GhBEL1-like members to form the heterodimers to regulate the downstream targets, and this regulatory relationship is partially conserved with *Arabidopsis*. In summary, this study provides important clues for further elucidating the functions of TALE genes in regulating cotton growth and development, especially in the fiber SCW biosynthesis network, and it also contributes genetic resources to the improvement of cotton fiber quality.

## Background

Cotton (*Gossypium hirsutum* L.) is one of the most important economic crops in the world because its natural textile fibers are the main resource for the textile industry. Cotton fibers are highly elongated and thickened single cells derived from the ovule epidermis and are also a powerful model systems for studying cell elongation and secondary cell wall (SCW) biosynthesis [1]. Fiber development includes four distinct and overlapping stages: initiation, elongation (primary cell wall (PCW) biosynthesis), SCW thickening (cellulose biosynthesis), and maturation. Fiber initiation starts 2 days before anthesis, and fibers enter the elongation phase immediately until approximately 21 days post anthesis (DPA), rapid and remarkable elongation of fiber cells is accompanied by a large number of PCW components (including crystalline cellulose fibrils, xyloglucan and pectin, etc.) synthesized [2]. The SCW thickening stage initiates at approximately 16 DPA, and cellulose is abundantly synthesized and deposited orderly on PCW at this stage, which determines the quality and yield of cotton fiber [3]. After 45 DPA, fiber cells enter a period of dehydration and maturation. In mature fibers, the 95% of the final dry weight can be attributed to cellulose [4]. Fiber length and strength are both key traits of fiber quality. Investigation of different cotton cultivars shows that fiber length is largely determined by the duration of the elongation stage, and fiber strength (FS) is tightly correlated with SCW biosynthesis and the array of crystal cellulose.

It is believed that the regulation of cotton fiber development requires a large number of transcription factors (TFs) and structural genes. In recent years, some genes involved in the regulation of early fiber development have been reported. For example, the R2R3-MYB transcription factors *GhMYB25* and *GhMYB25-like* regulate fiber initiation and elongation [5]. GhJAZ2 negatively regulates cotton fiber initiation by interacting with the R2R3-MYB transcription factor GhMYB25-like [6]. A putative homeodomain leucine zipper (HD-ZIP) transcription factor, *GhHD-1*, is expressed in trichomes and early fibers, and in ovules, it acts downstream of *GhMYB25-like* and plays a significant role in cotton fiber initiation [7]. *GhHOX3* from the class IV HD-ZIP family, which can interact with *GhHD1*, also showed strong expression during early fiber elongation [8]. The complex regulation of the early fiber development affects the final fiber density and length, while the regulation of the orderly deposition of cellulose during the secondary wall thickening stage affects the strength and flexibility of plants [1]. Many TFs related to cotton fiber initiation and elongation development have been identified and constitute a complex regulatory network involving a considerable number of members. So far, however, only a few proteins have been found to be involved in the synthesis of cotton fiber SCW, especially transcription factors. Two members of a new group of chitinase-like (CTL) group proteins, GhCTL1 and GhCTL2, have preferential expression during secondary wall deposition and are essential for cellulose synthesis in primary and secondary cell walls [9].. Brill et al. (2011) identified and characterized a novel Sus isoform (SusC) that was upregulated during secondary wall cellulose synthesis in cotton fiber [10]. Subsequently, overexpression of *GhSusA1* increased fiber length and strength, with the latter indicated by the enhanced thickening of the cell wall during the secondary wall formation stage [11]. The plant cell wall can regulate cell growth, provide structural and mechanical support for plants, and act as a barrier to the environment and potential organisms, which is based on its complex and dynamic structure [12]. After the cessation of cell growth, SCW is deposited inside the lignocellular or tracheal element cells in the PCW. Unlike the SCW of other plant cells, the cotton fiber SCW contains few noncellulosic components and little or no lignin, and lignification is transcriptionally repressed during cotton fiber SCW deposition [13]. Nevertheless, the main viewpoint on the regulation of lignocellulosic SCW biosynthesis is that a series of SCW-specific NAC and MYB TFs as the master switches regulate other downstream TFs including other NACs, MYBs and KNATs (knotted-like from *Arabidopsis thaliana*), and the SCW structural components biosynthetic genes which encoding cellulose synthases (CESAs), hemicellulose synthases and lignin-related enzymes are the main targets of TFs [14–16]. Although some TFs have been identified to be involved in the biosynthesis of SCW during plant growth and development, little is known about the characteristics of TFs in regulating the specific cotton fiber SCW formation. Characterizing these TFs related to SCW biosynthesis of cotton fiber cells will enable further understanding of the molecular mechanism of fiber development and improve cotton fiber quality by genetic manipulation.

The article "Genome-wide identification and characterization of TALE superfamily genes in cotton reveals their functions in regulating secondary cell wall biosynthesis" was retracted in 2024. Reasons: duplicated images; original data or images not available; unreliable results or conclusions; concerns about the data.

Members of the three-amino-acid-loop-extension (TALE) homeodomain superclass of homeoproteins contain a three-amino acid extension in the loop connecting the first and second helices of their homeodomain and comprise the KNOTTED-like homeodomain (KNOX) and BEL1-like homeodomain (BLH/BELL) proteins, which function as heterodimers that are structurally and functionally related. The plant TALE homeodomain superclass controls meristem formation and maintenance, organ morphogenesis, organ position, and several aspects of the reproductive phase [17]. The *Arabidopsis* KNOX family genes divided into three classes according to the similarity of homeodomain certain residues, intron positions, and expression patterns [18, 19]. Class I KNOX genes, including *STM*, *KNAT1/BP*, *KNAT2*, and *KNAT6* in *Arabidopsis*, play the role of transcriptional activation or repression in meristem development, leaf shape control, and hormone homeostasis [20–22]. The expression patterns and functional characteristics of the class II KNOX genes also show a wide range of diversity. For example, previous studies have shown that *KNAT3*, *KNAT4*, and *KNAT5* exhibit cell-type-specific expression patterns during the regulation of root development in *Arabidopsis* [23]. *AtKNAT7* and its homologous *PoptrKNAT7* negatively regulate SCW formation in *Arabidopsis* and *Populus*, respectively [24]. AtKNAT7 also can form a functional complex with MYB75 to modulate SCW deposition in both stems and seed coats [25]. *KNATM*, the only class III KNOX member, is involved in the regulation of leaf polarity, leaf shape and compound leaf development [26]. In *Arabidopsis*, all the 13 BEL1-like family members can form heterodimers with KNOX proteins [27]. The BEL1-like homeodomain (BLH) proteins are critical for meristem and floral development, and their functions are always overlapping and redundant. For example, *AtBLH1* controls the switch between synergistic cells and oocytes in the embryo sac [28]. The loss of *AtBEL1* gene function hinders the development of integuments [29]. SAW1 (BLH2) and SAW2 (BLH4) negatively regulated BREVIPEDICELLUS (BP/KNAT1), and *saw1saw2* double mutant leaves grew serrated and revolute, but they were positive regulators of growth [27]. AtBLH6 and AtKNAT7 interact and regulate SCW formation via repression of *REVOLUTA* [30]. *Arabidopsis thaliana* HOMEOBOX 1 (ATH1), PENNYWISE (PNY/BLH8), and POUNDFOOLISH (PNF/BLH9) play important roles in regulating the development of the shoot apical meristem and inflorescence architecture [31–33]. In crops, GmBLH4 might heterodimerize with GmSBH1 to form functional complexes and function in modulating plant growth and development as well as in response to high temperature and humidity stress in soybean [34]. Overexpression of *OsBLH6* and *OsSND1* leads to ectopic deposition of lignin and cellulose, and *OsBLH6* may function as SCW-associated TFs by enhancing the transcription of cell wall biosynthesis genes in rice [35]. In summary, TALE superfamily genes tend to exhibit functional conservatism in both crop and model plant *Arabidopsis*.

The article "Genome-wide identification and characterization of TALE superfamily genes in cotton reveals their functions in regulating secondary cell wall biosynthesis" was retracted in 2024. Reasons: duplicated images; original data or images not available; unreliable results or conclusions; concerns about the data.

A few gene function studies of cotton TALE members have been reported in recent years: *GhKNL1*, a homolog of *AtKNAT7* and encoding a class II KNOX protein, was reported to participate in regulating fiber SCW development of cotton [36], and *GhFSN1*, a homolog of *AtNST1*, was reported to function as an upstream regulator of *GhKNL1* to facilitate cotton fiber SCW deposition [37]. Despite these studies, our understanding of the TALE superfamily members in cotton is still very limited, and the role and position of TALE superfamily members in the cotton fiber SCW biosynthesis regulatory network is almost unknown. If any other KNOX members are involved in the regulation of the cotton fiber SCW biosynthesis and as the partner of the KNOX family proteins, the number and identity of BEL1-like family members participating in the regulation of SCW biosynthesis are still unknown. The genome sequences of two allotetraploid cotton species, *Gossypium hirsutum* - AD1 (upland cotton) and *Gossypium barbadense* - AD2 [38–41], and the two diploid species, *Gossypium raimondii* - D5 and *Gossypium arboreum* - A2 [42–44], provide an important genomic resource for a genome-wide analysis of the TALE gene family and other genetic and functional genomics studies.

In this study, 94 genes encoding TALE proteins were identified in upland cotton, including 44 KNOX family members and 50 BEL1-like family members, which is similar to the quantity found in *Gb* and twice the quantities found in *Ga* and *Gr*. Comparison of the characteristics and the expression pattern of upland cotton TALE family members revealed common and divergent features of the TALE family and may provide some clues about the function of the TALE genes. The chromosome colocalization of TALE family members with the FS-related quantitative trait loci (QTLs) narrowed our selection range for the TALE members participating in the regulation of cotton fiber SCW formation, and combined with the expression patterns of the candidate TALE members in different fiber quality materials, we believe that GhKNAT7 homologous genes may be the only KNOX subgroup members and play a key role in the regulation of SCW biosynthesis by mainly suppressing lignin synthesis. Yeast two-hybrid (Y2H) assays revealed that some BEL1-like members also function in regulating SCW biosynthesis by interacting with GhKNAT7, which was also identified by transgenic assays in *Arabidopsis*. A cis-element analysis and yeast one-hybrid (Y1H) assays identified the regulatory relationships between TALE members and other TFs such as *GhMYB46* and some genes encoding SCW biosynthetic enzymes in the network of cotton SCW biosynthesis regulation. In summary, the identified TALE proteins could form heterodimers or even polymers to perform their function in cotton fiber development, they are direct targets of some upstream TFs and could also directly regulate the expression of some genes encoding SCW biosynthetic enzymes. This arrangement is similar to that in *Arabidopsis*, except for some potential cotton species-specific BEL1-like members such as GhBEL1*,* GhBLH2, GhBLH4 and GhBLH7 subgroup members, which may also function as midstream regulators in the cotton fiber SCW biosynthesis network. Our results provide the molecular function and regulation of TALE family genes in cotton FS formation and provide a theoretical basis for cotton breeding.

The article "Genome-wide identification and characterization of TALE superfamily genes in cotton reveals their functions in regulating secondary cell wall biosynthesis" was retracted in 2024. Reasons: duplicated images; original data or images not available; unreliable results or conclusions; concerns about the data.

## Results

### Genome-wide identification of the TALE transcription factor superfamily genes in four *Gossypium* species

To identify all of the TALE proteins in *G. hirsutum* and *G. barbadense* (AADD genome) and its two diploid ancestors, *G. arboreum* (AA genome) and *G. raimondii* (DD genome), we used the *Arabidopsis* TALE protein sequences to match the four reference genomes to screen candidate TALE-like proteins in cotton. After a strict two-step selection process, 46 deduced TALE superfamily genes were identified in *G. arboreum*, along with 47 in *G. raimondii*, 88 in *G. barbadense* and 94 in *G. hirsutum*, based on gene homology, and all of the TALE superfamily members can be clearly divided into two groups, the BEL1-like family and KNOX family (Fig. 1a,c). Among the genes of the four *Gossypium* species, 24, 25, 46 and 50 genes belong to the BEL1-like family and 22, 22, 42 and 44 members belong to the KNOX family, respectively. It is noteworthy that compared with *A. thaliana*, there were no members in *Gossypium* species homologous to BLH3, BLH10 and KNAT5 (Fig. 1c, Additional file 4: Table S1).

**Fig. 1:** Phylogenetic and evolutionary analysis of TALE superfamily genes in four *Gossypium* species and *Arabidopsis thaliana*. **a** Phylogenetic analysis of these genes in four *Gossypium* species. **b** The ratio of nonsynonymous to synonymous substitutions (Ka/Ks) of TALE genes in *G. hirsutum* (AD1, AtDt), *G. barbadense* (AD2, AtDt), *G. raimondii* (D5), and *G. arboreum* (A2). **c** Number of TALE genes in the four *Gossypium* species and *A. thaliana*. A phylogenetic tree was constructed by MEGA 6.0 software using the neighbor-joining (NJ) method

We also explored the molecular evolutionary properties of TALE genes in all four *Gossypium* species. The calculation of substitution rates of nonsynonymous (Ka) and synonymous (Ks) can help us understand the evolutionary dynamics and selection pressures of protein-coding sequences. The relationship between Ka/Ks ratio and value 1, i.e. Ka equals Ka (Ka/Ks = 1), Ka less than Ks (Ka/Ks < 1) and Ka larger than Ks (Ka/Ks > 1), which represent neutral mutation, negative (or purifying) selection and positive (or diversifying) selection respectively. Most of the Ka/Ks ratios of the TALE gene pairs were less than 1 in the intergenomic (At and Dt or A2 and D5) and intragenomic (A2 and At or D5 and Dt) comparisons, except for 16 paired genes (Additional file 5: Table S2). The results suggested that purifying selection of most TALE genes in both diploid and allotetraploid cotton species occurred, and the fact that the Ka/Ks ratios of some pairs of genes are greater than 1 suggest that these genes may have played a key role in the evolution of allotetraploid *G. hirsutum* and *G. barbadense*. Furthermore, the average Ka/Ks values were higher in intragenomic comparisons than in the intergenomic comparisons, and the KNOX family had higher average Ka/Ks values than the BEL1-like family in upland cotton; however, the opposite was observed in *G. barbadense* (Fig. 1b), which may imply that evolutionary selection for the two families differed between these two cotton species.

The article "Genome-wide identification and characterization of TALE superfamily genes in cotton reveals their functions in regulating secondary cell wall biosynthesis" was retracted in 2024. Reasons: duplicated images; original data or images not available; unreliable results or conclusions; concerns about the data.

### Phylogenetic analysis and classification of TALE transcription factors

Systematic classifications of cotton TALE TFs at a genome-wide level have not been reported. To gain further insights into the evolutionary relationships, we employed MEGA 6.0 software to construct an unrooted phylogenetic tree of TALE members from *G. raimondii*, *G. arboreum*, *G. hirsutum*, *G. barbadense* and *A. thaliana*. The phylogenetic tree clearly showed that the TALE superfamily genes were clustered into two families (BEL1-like and KNOX family), so we constructed an unrooted phylogenetic tree for BEL1-like family genes and KNOX family genes seperately to better understand their evolutionary relationships (Fig. 2a, b). Based on the classification of *A. thaliana* TALE superfamily (BEL1-like and KNOX family) proteins, the *Gossypium* BEL1-like proteins were classified into 5 subfamilies (tuberization and root growth, leaf morphology, OFP (ovate family protein) partners, meristem function and ovule morphology) (Fig. 2a), and the KNOX proteins were divided into 3 subfamilies (class I, class II and class III) (Fig. 2b) [17, 45].

**Fig. 2:** Phylogenetic analysis and classification of BEL1-like and KNOX family genes in four *Gossypium* species and *Arabidopsis thaliana*. **a** Phylogenetic analysis and classification of BEL1-like family genes. **b** Phylogenetic and classification analysis of KNOX family genes. The subfamilies of the BEL1-like and KNOX members are represented by different colors. Numbers on the branches are bootstrap proportions of 1000 replicates. *Ga*, *Gossypium arboreum*; *Gr*, *Gossypium raimondii*; *Gh*, *Gossypium hirsutum*; *Gb*, *Gossypium barbadense*; *At*, *Arabidopsis thaliana*. The phylogenetic tree was constructed by MEGA 6.0 software using the neighbor-joining (NJ) method

The progenitors of *G. arboreum* (A2) and *G. raimondii* (D5) are the putative donors of the At and Dt subgenomes to the world-wide fiber-producing cotton species *G. hirsutum*, which is allotetraploid. Our phylogenetic results also supported the above finding, with orthologs from A (A2, At) genomes or D (D5, Dt) genomes exhibiting closer phylogenetic relationships than reciprocal comparisons between A (A2, At) and D (D5, Dt) genomes. Furthermore, some TALE homologous genes were missing in some *Gossypium* species, such as the homologs of *GhBLH7-A06*, *GhBLH8-A03* and *GhBEL1-A12* which were absent in the At subgenome of *G. barbadense*, but *GhBLH6-A12* had two homologs. Additionally, class III KNOX member *KNATM* homologs are present in both the At and Dt subgenomes of allotetraploid cottons and the diploid *G. raimondii* genome, which might be a gene lost in the A genome donor, *G. arboreum* (Additional file 4: Table S1). In addition to the deletion or replication of individual homologs in different *Gossypium* species, most genes were stable among the four species, which to some extent indicates that TALE genes may be functionally conserved between model plants, cotton crops and even cotton ancestor species.

### Structural analysis of TALE transcription factors in upland cotton

Since the analyses of gene structure could help us understand gene functions, regulation, and evolution [46], the structure of GhTALE genes in upland cotton was also identified. To better understand the evolutionary relationships between different members of the GhTALE superfamily, we first constructed two separate unrooted phylogenetic trees with GhBEL1-like and GhKNOX family gene DNA sequences, respectively (Fig. 3a, Additional file 1: Figure S1a). To elucidate the structural features of GhTALE genes, the gene exon/intron structures and the protein motifs structures of GhBEL1-like and GhKNOX family genes were analyzed, respectively (Fig. 3b-c, Additional file 1: Figure S1b-c).

The article "Genome-wide identification and characterization of TALE superfamily genes in cotton reveals their functions in regulating secondary cell wall biosynthesis" was retracted in 2024. Reasons: duplicated images; original data or images not available; unreliable results or conclusions; concerns about the data.

**Fig. 3:** Phylogenetics, gene structure, motif analysis, promoter cis-elements and expression patterns of GhBEL1-like genes. **a** Phylogenetic relationships of BEL1-like members of upland cotton and *A. thaliana*. The phylogenetic tree (left panel) was constructed with MEGA 6.0 using the neighbor-joining (NJ) method with 1000 bootstrap replicates. **b** Gene structure analysis of GhBEL1-like and AtBEL1-like genes. Gene structure maps were drawn with the Gene Structure Display Server 2.0. The scale bar is shown at the bottom. **c** Motif analysis of GhBEL1-like and AtBEL1-like proteins. All motifs were identified by MEME software (http://meme-suite.org/). The lengths of each motif are shown proportionally. **d** Cis-element analysis of GhBEL1-like gene promoters. The cis-elements were identified by PlantCARE software for the 1.5 kb upstream from the start codon of GhBEL1-like genes. **e** The expression patterns of GhBEL1-like genes in various tissues: root, stem, leaf, tours, ovules (− 3 to 3 DPA) and fibers (5 to 25 DPA). The FPKM values of TM-1 RNA-Seq data were used to construct the heatmap

The number of exons ranged from 1 to 7, with an average of 4.86 for all GhTALE members. The GhBEL1-like family genes mostly contained 4 exons, except for *GhBLH8-A10/D10*, which has only one exon; two pairs of orthologous genes, *GhBEL1-A/D12* and *GhBLH9-A/D10,* which have 3 exons; and *GhBEL1-D03* and *GhBLH6-D02*, which have different numbers of exons with their At subgenome homologs, which contain 5 and 7 exons, respectively (Fig. 3b). In comparison, the GhKNOX family mainly comprised 5 exons, and the number of exons ranged from 3 to 6. Specifically, the *GhSTM* subgroup genes always have 4 exons, which is the same number as the *Arabidopsis* homologous gene, *AtSTM*; while the class III KNOX subfamily *GhKNATM* genes have 3 exons, which are different from their *Arabidopsis* homologous gene, *AtKNATM* (Additional file 1: Figure S1b). These results reveal that gene structures generally exhibited a highly conserved distribution of exons and introns within the same phylogenetic subfamily or subgroup in upland cotton.

In general, both BEL1-like and KNOX proteins contain a TALE homeodomain (also called a homeobox domain, which always shares sequence with a Homeobox_KN domain), While BEL1-like proteins harbor a POX (also named MID) domain composed of the SKY and BELL regions, and KNOX proteins contain a MEINOX domain composed of two subdomains (KNOX1 and KNOX2) separated by a flexible linker and an ELK domain. The BELL region of BEL1-like proteins interact with MEINOX domain of KNOX proteins mediates the formation of heterodimers. Among the 94 GhTALE proteins, the lengths of the identified GhBEL1-like proteins ranged from 164 (GhBLH8-A10) to 817 (GhBLH2-A11) amino acids (aa), with an average length of 473 aa, and GhBLH8-A/D10 homologous proteins only have a shorter POX domain and lacked the homeobox domain (Fig. 3c). Meanwhile, the GhKNOX proteins ranged from 161 (GhKNATM-A/D12 homologs) to 681 (GhKNAT3-A13) aa, with an average length of 495 aa. The class III KNOX KNATM protein has no homeodomain, which is the same arrangement as its *Arabidopsis* homolog. All GhKNOX members contain the KNOX1 and KNOX2 (MEINOX) domain conservatively, but some proteins deleted from other domains, such as GhKNAT2-A08 and GhKNAT6-D05 were missing the homeobox domain, and GhKNAT4-A06 was missing both the ELK and homeobox domains. Interestingly, GhKNAT7-A/D12 homologs have one ELK domain more than their paralogous genes GhKNAT7-A/D03 and GhKNAT7-A/D08, which may lead to the differentiation of functions in the subgroups (Additional file 1: Figure S1c).

The article "Genome-wide identification and characterization of TALE superfamily genes in cotton reveals their functions in regulating secondary cell wall biosynthesis" was retracted in 2024. Reasons: duplicated images; original data or images not available; unreliable results or conclusions; concerns about the data.

### Cis-element analysis and expression patterns of GhTALE transcription factors

Transcriptional control is an important method of regulating gene expression, and cis-acting elements play a key role in this process. Among the cis-elements identified, we mainly chose phytohormone-related elements, transcription factor binding sites and those involved in abiotic stress responses for analysis. A total of 25 types of putative candidate cis-elements were present in the promoters of GhTALEs (Fig. 3d, Additional file 1: Figure S1d), and gibberellin (GA)- and salicylic acid (SA)-related elements (P-box, TATC-box, GARE-motif and TCA-element), MYB transcription factor binding sites (MBSI, MBSII and MBS) and as-2-box elements were the most abundant of the three selected types of cis-acting elements (Additional file 2: Figure S2a). This result suggests the important roles of GhTALE genes in biological processes as well as in responses to phytohormones and abiotic stresses in cotton.

Notably, cis-elements involved in hormone responsiveness were distributed in almost all GhTALE gene promoters, which shows that the TALE genes may be involved in many processes of cotton growth and development, similarly to their roles in *Arabidopsis*. Specifically, the numbers and locations of the hormone-related cis-elements showed great variance among different GhTALE genes. For example, only one type of IAA-related cis-element (TGA-element) was present in the *GhKNAT1-A02* promoter, but cis-elements related to all five hormones (abscisic acid (ABA), indole-3-acetic acid (IAA), GA, SA and jasmonate (JA)) were present in the promoter of *GhKNAT7-A12*. There were no ABA-related cis-elements in the GhKNAT1 and GhKNAT3 subgroup promoters. Furthermore, the distribution of the phytohormone-related cis-elements varied even in the promoters of the GhBEL1-like or GhKNOX genes clustered in the same subgroup, which is in sharp contrast to the sequence conservation shown in the coding region of the same subgroup genes. As in the GhKNAT7 subgroup, *GhKNAT7-A/D08* promoters contained only one type of SA-related elements (TCA-element), but *GhKNAT7-A/D03* and *GhKNAT7-A/D12* promoters contained 8 kinds of cis-elements related to all five hormones (Additional file 8: Table S5). This result suggests that TALE genes in the same subgroup may participate in different growth and development processes through producing specific tissue expression patterns or differential expression regulation.

The article "Genome-wide identification and characterization of TALE superfamily genes in cotton reveals their functions in regulating secondary cell wall biosynthesis" was retracted in 2024. Reasons: duplicated images; original data or images not available; unreliable results or conclusions; concerns about the data.

Previous studies have suggested that TALE genes are expressed in all plant tissues and are regulated temporally and spatially depending on environmental conditions and developmental stage. Recently published research reported *G. hirsutum* acc. TM-1 gene expression profiles, including those in 10 different types of tissues and organs, which allowed us to investigate the expression of GhTALE family members in different organs and developmental stages [39]. We selected 4 organs (root, stem, leaf and torus) and 9 ovule and fiber developmental stages (− 3 to 3 DPA ovules, and 5 to 25 DPA fibers) for constructing the expression heatmaps of GhBEL1-like and GhKNOX genes (Fig. 3e and Additional file 1: Figure S1e). The FPKM (fragments per kilobase of exon per million fragments mapped) method was employed to normalize the total short read sequences, and all of the 94 GhTALE genes had an FPKM > 1 in at least one of the 13 investigated samples. Among the 44 GhKNOX genes, only the class II KNOX subfamily *GhKNAT7* subgroup homologs showed significantly dominant expression in the SCW thickening period, but in the GhBEL1-like genes, *GhBEL1*, *GhBLH1*, *GhBLH2*, *GhBLH4*, *GhBLH5*, *GhBLH6*, *GhBLH7* and *GhBLH9* subgroups had relatively high expression levels at 20 and 25 DPA. These data suggested that these GhTALE members might participate in the regulation of cotton fiber development, especially at the SCW biosynthesis stage. Meanwhile, *GhKNAT1* homologs were showed significant dominant expression in leaf tissue, which may play a remarkable role in regulating leaf development. In addition, *GhKNAT3* and *GhKNAT4* were highly expressed in torus, and *GhSTM* and *GhKNAT6* were highly expressed in both root and leaf. In contrast to GhKNOX members, which showed distinct tissue specificity, GhBEL1-like members always exhibited high expression in several tissues; for example, *GhBEL1*, *GhBLH2*, and *GhBLH4* subgroup genes were strongly expressed in stem and torus. *GhBLH1* and *GhBLH5* genes were highly expressed in various tissues and organs (including leaf, root, stem and torus). *GhBLH6* and *GhBLH7* were highly expressed in stem, while all of the GhBEL1-like genes mentioned above also displayed high expression in fiber SCWs. In addition, *GhBLH8* and *GhBLH9* members were specifically highly expressed in root and leaf. Differences in TALE family gene expression patterns also reflect their diversity in regulating cotton growth and development. It is clear that many BEL1-like and KNOX family genes play important roles in the regulation of cotton fiber SCW biosynthesis.

The article "Genome-wide identification and characterization of TALE superfamily genes in cotton reveals their functions in regulating secondary cell wall biosynthesis" was retracted in 2024. Reasons: duplicated images; original data or images not available; unreliable results or conclusions; concerns about the data.

Phytohormones play an important role in various biological functions when plant tissues and organs develop or when they are subjected to abiotic stresses. We also explored the expression of GhTALE genes in response to GA and SA. Due to the high similarity between the nucleotide sequences of the homologous genes, we designed 8 pairs of primers specific for each of the selected homologous genes to detect their expression by qRT-PCR. Our results showed that the transcript levels of some selected genes such as *GhKNAT7*, *GhBEL1*, *GhBLH1* and *GhBLH6* homologs responded to GA and SA. It is remarkable that even the paralogous genes respond differently to the hormones. For example, *GhKNAT7-A/D08* are significantly induced by SA but inhibited by GA compared with the control, while *GhKNAT7-A/D12* are inhibited by both SA and GA. *GhKNAT7-A/D03* are inhibited by the hormones in the early stage of treatment (e.g., 1 to 3 h after the treatment), and then reversed increased (Additional file 2: Figure S2b), suggesting that GhTALE genes participate in the regulation of GA and SA signal transduction, that the expression of these GhTALE genes may be regulated by a large number of TFs and signaling molecules upstream and that there may also be feedback regulation in the GhTALE protein regulation pathway. More interesting is that some BEL1-like members responded to SA and GA are consistent with *GhKNAT7* homologs, such as the response of *GhBLH1-A/D01* to hormones is similar to that of *GhKNAT7-A/D03*, *GhBLH6-A/D03* and *GhBEL1-A/D03* are consistent with *GhKNAT7-A/D08* and *GhKNAT7-A/D12*, respectively. These results suggest that GhBEL1-like members may take functions simultaneously with GhKNOX members in regulating cotton growth and development.

The article "Genome-wide identification and characterization of TALE superfamily genes in cotton reveals their functions in regulating secondary cell wall biosynthesis" was retracted in 2024. Reasons: duplicated images; original data or images not available; unreliable results or conclusions; concerns about the data.

### Identification of SCW-associated TALE superfamily members by chromosome colocalization analysis and differential expression analysis

The 94 GhTALE genes were located on all 26 chromosomes in *G. hirsutum* acc. TM-1, with an equal number distribution of 47 genes (25 GhBEL1-like genes and 22 GhKNOX genes) on both the At and Dt subgenome chromosomes. However, they were unevenly distributed on each chromosome, and the homologous chromosomes At/Dt01, At/Dt04, At/Dt09, and At/Dt11 contained two pairs of GhTALE genes on themselves, respectively. Six pairs of GhTALE genes were located on both At/Dt06 and At/Dt12, and At/Dt05 had eight pairs of GhTALE homologs on them.

To reveal if these GhTALE genes are genetically involved in fiber SCW development, we performed a genome-wide colocalization analysis of all GhTALE TFs in all 26 chromosomes of the sequenced TM-1 genome with fiber SCW-related trait QTLs in intraspecific upland populations and interspecific *G. hirsutum* × *G. barbadense* populations from CottonQTLdb (www.cottonqtldb.com). The two fiber SCW traits were FS and wall thickness (WT). There were 330 and 110 FS QTLs in intraspecific upland populations and interspecific *G. hirsutum* × *G. barbadense* populations, respectively, and they were downloaded for analysis, and 13 WT QTLs were found in only intraspecific upland populations (Additional file 6: Table S3). The genome-wide analysis identified 14 GhKNOX genes and 21 GhBEL1-like genes that were colocalized with fiber SCW-related trait QTL hotspots (containing at least four QTLs for the same trait within a 20-cM region, as defined by Said et al.) on different chromosomes [47–49]. Coincidently, five of the six *GhKNAT7* homologs were among the 14 GhKNOX genes, in addition to 3 *GhKNAT2*s, 2 *GhKNAT1*s, 2 *GhSTM*s, 1 *GhKNAT3* and 1 *GhKNATM*. The 21 candidate GhBEL1-like genes included 5 *GhBLH5*s, 3 *GhBEL1*s, 3 *GhBLH1*s, 3 *GhBLH8*s, 2 *GhBLH9*s, 2 *GhBLH11*s, 1*GhBLH6*, 1 *GhBLH7* and 1 *GhATH1* (Fig. 4a-b, Additional file 3: Figure S3). These results, to a certain extent, were partly consistent with the expression pattern analysis for candidate GhTALE members involved in SCW biosynthesis regulation.

**Fig. 4:** A genome-wide analysis of colocalization of all GhTALE genes in the sequenced genome TM-1 chromosomes (A08 and A12) with QTL hotspots for fiber strength (FS) and wall thickness (WT) traits in intraspecific upland cotton populations and interspecific *G. hirsutum* × *G. barbadense* populations. **a** QTL colocalization analysis of GhTALE genes on the A08 chromosome. **b** QTL colocalization analysis of GhTALE genes on the A12 chromosome. Gray shadowed segments indicate the QTL clusters on chromosomes. The range covered by black solid lines indicates the QTLs in the hotspot on chromosomes. The dotted line indicates the GhTALE genes in the QTL regions (but not at a hotspot or cluster) on chromosomes

In addition, four other genes (*GhFSN1*, *GhFSN2*, *GhMYB46/83*, and *GhKNL1*) that were reportedly related to fiber SCW development were colocalized with the FS-related QTLs on corresponding chromosomes, which means that the colocalization analysis for candidate genes of related traits is reliable (Fig. 4a-b, Additional file 3: Figure S3).

The article "Genome-wide identification and characterization of TALE superfamily genes in cotton reveals their functions in regulating secondary cell wall biosynthesis" was retracted in 2024. Reasons: duplicated images; original data or images not available; unreliable results or conclusions; concerns about the data.

Based on the QTL chromosome colocalization and the transcriptome data sets, GhKNAT7 homologs and some BEL1-like family members were selected for verifying the expression changes during fiber development (10, 20 and 30 DPA) in three upland cotton varieties (Suyou 6018, TM-1, Ken 27) with different fiber quality by qRT-PCR (Fig. 5a). The different expression levels of CESA4 and CESA8 were consistent with the FS quality of the three selected varieties, while Suyou 6018 had the highest FS and the highest expression of *GhCESA4* and *GhCESA8* during fiber SCW biosynthesis (20 and 30 DPA). Ken 27 had the least of these values (Fig. 5b). Because the main component of the cotton fiber SCW is cellulose, the expression patterns of lignin synthesis-related genes in the three varieties were the opposites of those of cellulose synthesis-related genes, and *GhCAD5* and *GhCOMT1* expressed at higher levels in cultivars with low FS than in those with high FS. Except for *GhBLH5-A/D07*, which was dominant expression at 10 DPA, other GhTALE members were predominantly expressed during the critical period of SCW biosynthesis. These expression data were the same as the transcriptome data, and these members tended to have higher transcriptional levels in high-FS varieties than in low-FS varieties. These results suggest that GhTALE superfamily genes may promote the synthesis of cellulose and inhibit the synthesis of lignin during the thickening of the fiber SCW, thus creating a favorable environment for high levels of cotton FS formation.

**Fig. 5:** Analysis of the expression patterns of GhTALE genes and cellulose and lignin biosynthesis-related genes during fiber development (10, 20 and 30 DPA) in three upland cotton varieties with different fiber quality by qRT-PCR. **a** The fiber length and fiber strength of three upland cotton varieties. **b** Expression profiling of fiber SCW biosynthesis-related candidate GhTALE genes and cellulose and lignin biosynthesis-related genes during fiber development. Gene expression data were obtained by quantitative real-time PCR with three independent replicates

The article "Genome-wide identification and characterization of TALE superfamily genes in cotton reveals their functions in regulating secondary cell wall biosynthesis" was retracted in 2024. Reasons: duplicated images; original data or images not available; unreliable results or conclusions; concerns about the data.

### GhKNAT7 and GhBLH6 influence the stem morphological structure and chemical composition in transgenic *Arabidopsis*

In the model plant *A. thaliana*, the TALE family members AtBLH6 and AtKNAT7 interact and regulate SCW formation via repression of *AtREV* [30]. It has been indicated that cotton fiber SCW formation is similar to the corresponding process in the *Arabidopsis* xylem [50]. Therefore, *Arabidopsis* was employed for investigating the role of GhTALE genes in the regulation of SCW formation. *GhKNAT7* and *GhBLH6* overexpression constructs (35S:*GhKNAT7-A03* and 35S:*GhBLH6-A13*, respectively) were introduced into *Arabidopsis*. Over 10 lines of both 35S:*GhKNAT7-A03* and 35S:*GhBLH6-A13* transgenic *Arabidopsis* were obtained, and at least four lines (generation T_3_) were selected for further study. A comparison of the phenotypes of wild-type and transgenic plants clearly showed fascicular stems in a percentage of both 35S:*GhKNAT7-A03* and 35S:*GhBLH6-A13* transgenic plants. Otherwise, wild-type Col-0 plants displayed normal morphology in basal stems (Fig. 6a). Additionally, histological staining showed that the SCW thickness of interfascicular fibers was significantly decreased in both *35S:GhKNAT7-A03* and *35S:GhBLH6-A13* transgenic plants. Nevertheless, the SCW of xylem fibers and vessels in the transgenic lines was almost unchanged compared with the wild type (Fig. 6b). The cell WT of interfascicular fibers was 1.72 ± 0.18 μm and 2.09 ± 0.25 μm in *35S:GhKNAT7-A03* and *35S:GhBLH6-A13* plants, respectively, while it was 2.76 ± 0.22 μm in wild type (*n* > 20 cells for each individual line, total of four lines for each of the transgenes measured) (Fig. 6c), which further validated the inhibitory effects of cotton TALE TFs on lignin biosynthesis and the idea that TALE genes may influence the shape of the SCW and further affect stem morphology in *Arabidopsis*.

**Fig. 6:** Phenotypes of 35S:*GhKNAT7-A03* and 35S:*GhBLH6-A13* transgenic *Arabidopsis* plants. **a** Phenotypes of wild-type, 35S:*GhKNAT7-A03* and 35S:*GhBLH6-A13* transgenic *Arabidopsis* plants. Phenotypes were observed in six-week-old seedlings. **b** Phloroglucinol-HCl staining of stem cross-sections of wild-type, 35S:*GhKNAT7-A03* and 35S:*GhBLH6-A13* transgenic *Arabidopsis* plants. **c** Comparison of SCW thickness of interfascicular fibers of wild-type, 35S:*GhKNAT7-A03* and 35S:*GhBLH6-A13* transgenic plants. Each experiment was performed in three biological replicates, and the error bars represent the mean ± SE. *P < 0.05; **P < 0.01. Scale bar = 1 cm in (**a**) and 10 μm in (**b**). If, interfascicular fiber

The article "Genome-wide identification and characterization of TALE superfamily genes in cotton reveals their functions in regulating secondary cell wall biosynthesis" was retracted in 2024. Reasons: duplicated images; original data or images not available; unreliable results or conclusions; concerns about the data.

### Interactions between GhBEL1-like and GhKNOX family members

In *Arabidopsis*, KNOX proteins interact with BEL1-like proteins, which are essential components for KNOX/BELL heterodimerization. The most representative example of this behavior is that AtKNAT7 interacts with AtBLH6 to regulate SCW formation in *A. thaliana* [30]. Based on the expression pattern analysis and the genome-wide QTL colocalization analysis of SCW-related GhTALE genes, we performed a large-scale Y2H experiment to systematically analyze the interactions between GhKNAT7 subgroup members and GhBEL1-like proteins. In total, 3 *GhKNAT7* subgroup members and 16 GhBEL1-like genes (including *GhBEL1*, *GhBLH1*, *GhBLH2*, *GhBLH4*, *GhBLH5*, *GhBLH6* and *GhBLH7* subgroup members) were cloned and sequenced to confirm their complete open reading frame (ORF), and then they were constructed into DNA-binding domain and activation domain plasmid vectors, respectively. Each BEL1-like/KNAT7 pair was individually cotransformed into Y2H yeast cells.

Interestingly, all members of GhBEL1, GhBLH1 and GhBLH6 subgroups can form heterodimers with all GhKNAT7 subgroup proteins, but some other proteins interact with only individual member proteins of the GhKNAT7 subgroup. For example, GhBLH5-D09 interacts with only GhKNAT7-A03 and GhKNAT7-D12 and not with GhKNL1 (GhKNAT7-D08). GhBLH5-D07 interacts with none of GhKNAT7 subgroup homologs (Fig. 7a). It is remarkable that the KNAT7/BLH6 and KNAT7/BLH5 pair interactions were previously reported in *Arabidopsis* and other crops [30, 51], and the former pair had well-defined functions in regulating SCW biosynthesis. The GhKNAT7/GhBEL1 and GhKNAT7/GhBLH1 pair interactions were newly discovered and may even be cotton species specific. These results suggest that the molecular mechanism of regulating fiber SCW thickening in cotton may be slightly different from that in *Arabidopsis* because of their differences in cell wall composition. GhKNAT7 proteins may participate in cotton fiber cell wall biosynthesis by interacting with more GhBEL1-like factors than homologous proteins of *Arabidopsis*, which also indicates the complexity of cotton fiber development regulation.

**Fig. 7:** The interaction between GhKNAT7 and selected GhBEL1-like members and the regulation relationship of TALE heterodimers. **a** Yeast two-hybrid assay (Y2H). DDO, yeast medium lacking leucine and tryptophan. QDO, yeast medium lacking leucine, tryptophan, histidine and adenine. 3-AT, 3-amino-1,2,4-triazole. **b** Putative TFBSs for GhMYB46 (M46-B1 and M46-B2) and GhKNAT7 (K7-B1 and K7-B2). **c** Expression heatmap of GhMYB46 homologs. **d** The selected GhMYB46 and GhKNAT7 TFBSs sequences on most predicted promoters of the GhTALE members and lignin and cellulose biosynthesis genes. **e** Yeast one-hybrid assay (Y1H). DDO, yeast medium lacking leucine and tryptophan. TDO, yeast medium lacking leucine, tryptophan, and histidine. 3-AT, 3-amino-1,2,4-triazole

The article "Genome-wide identification and characterization of TALE superfamily genes in cotton reveals their functions in regulating secondary cell wall biosynthesis" was retracted in 2024. Reasons: duplicated images; original data or images not available; unreliable results or conclusions; concerns about the data.

### The TALE homeoprotein heterodimers are regulated by GhMYB46 and directly regulate the expression of downstream SCW biosynthesis genes

We have identified the inhibitory effect of SCW-related GhTALE family members on lignin biosynthesis in *Arabidopsis* interfascicular fibers. To identify the role of TALE proteins in the cotton fiber SCW biosynthesis regulatory network, conserved promoter elements present in at least two different species (including *Arabidopsis* and cotton) were considered in the search for putative transcription factor binding sites (TFBSs). Previous studies have shown that the expression of *AtKNAT7* is directly regulated by AtMYB46 in *A. thaliana* [52]. Moreover, the cis-element analysis of TALE member promoters also showed that the MYB TF binding sites accounted for the greatest number of TFBSs, which implies an important role for MYB transcription factors in regulating TALE gene expression. Accordingly, PlantPAN 2.0 was used as a database for scanning of potential GhMYB46 and GhKNAT7 recognition sites in the predicted promoters of GhTALE family genes and the structural genes of the lignin and cellulose biosynthesis pathways [53]. We found that GhMYB46 and GhKNAT7 binding sites are present in predictive promoters of both numerous GhTALE members and lignin and cellulose biosynthesis pathway genes (Additional file 9: Table S6). For instance, *GhCAD5* and *GhCOMT1* both have expression trends that are the opposites of those of *GhKNAT7* homologs during fiber development, indicating that GhKNAT7 may directly inhibit their expression by binding to their promoters to regulate lignin biosynthesis and affect fiber SCW formation. Moreover, the promoters of many GhBEL1-like genes (including *GhBEL1*, *GhBLH1*, *GhBLH2*, *GhBLH5* and *GhBLH6* subgroup genes) and several *GhKNAT7* homologs (including *GhKNAT7-D03* and *GhKNAT7-D12*) also contained GhKNAT7-binding sites, which hinted that there may be a much feedback regulation between TALE TFs in addition to the interaction.

Y1H assays were used to confirm these upstream and downstream regulatory relationships and to identify the location of TALE homeoprotein heterodimers in the cotton fiber SCW biosynthesis regulatory network. First, the expression of all GhMYB46 homologs during fiber development was observed in the published transcriptome database, and *GhMYB46-A/D13* were predominantly expressed in the SCW thickening stage; their levels were also significantly higher than those of other homologs (Fig. 7c). Based on the TFBSs scanning of GhMYB46-A/D13 and GhKNAT7 members in PlantPAN 2.0, we selected two types of conserved cis-elements for each gene for the construction of the Y1H vectors (pHIS2) (Fig. 7b). The results confirmed that GhKNAT7 binds at the gtTGACAgca (K7-B1) and aTGTCAag (K7-B2) sites, which frequently appeared in the predicted promoters of the structural genes of the lignin and cellulose biosynthesis pathways and in some GhBEL1-like family member promoter regions. On the other hand, the promoter region of *GhKNAT7* homologs and some GhBEL1-like genes contained one or several gtTAGGTt (M46-B1) and cAACCAcc (M46-B2) sites, which can be bound by the upstream TFs GhMYB46-A/D13 to promote the expression of those *GhKNAT7* homologs and GhBEL1-like genes (Fig. 7d, e).

The article "Genome-wide identification and characterization of TALE superfamily genes in cotton reveals their functions in regulating secondary cell wall biosynthesis" was retracted in 2024. Reasons: duplicated images; original data or images not available; unreliable results or conclusions; concerns about the data.

## Discussion

During the past few years, the whole-genome sequences of four cotton species have been completed [38–44], and resequencing studies of large cotton varieties have also been performed, providing a good foundation for improving research on cotton functional genomics [54–57].

### TALE family members are highly conserved in structure and regulate SCW biosynthesis

In the present study, we reported for the first time the genome-wide identification of TALE superfamily genes (including BEL1-like and KNOX family members) and systematically investigated the functional structure of TALE TFs. We identified 46, 47, 94 and 88 TALE genes in *G. arboreum*, *G. raimondii*, *G. hirsutum* and *G. barbadense*, respectively (Additional file 4: Table S1). Depending on the phylogenetic and evolutionary analysis and the gene structure analysis of TALE genes, except for individual genes from the At/Dt subgenome that lack some protein motifs, such as GhKNAT2-A08, GhKNAT6-D05 and GhKNAT4-A06, most of GhTALE homeologous genes have closer evolutionary relationships and similar DNA and protein structures, even with their orthologous genes in diploid progenitors and *Arabidopsis*. The conservation of the homeobox domains among TALE repressors suggests a high level of functional redundancy in this family. In upland cotton, the expression patterns of GhTALE genes were comprehensively analyzed. We found that some homeologous genes had similar expression patterns, especially in the SCW thickening stage, also suggesting functional redundancy in the GhTALE gene family.

A cis-element analysis revealed that various hormone-responsive cis-elements appear on most of the GhTALE gene promoters, suggesting that the GhTALE proteins may respond to multiple phytohormone signals (Additional file 8: Table S5). Previous studies suggested that bioactive GAs promoted SCW deposition in cotton fibers by enhancing sucrose synthase expression [58]. Our study shows that some GhTALE genes respond to both GA and SA, which indicates that GhTALE genes may mediate the crosstalk between phytohormones and SCW biosynthesis regulation.

The article "Genome-wide identification and characterization of TALE superfamily genes in cotton reveals their functions in regulating secondary cell wall biosynthesis" was retracted in 2024. Reasons: duplicated images; original data or images not available; unreliable results or conclusions; concerns about the data.

Comparative analysis of gene expression patterns in materials with differences in fiber quality is a powerful approach for investigating genes involved in key stages of cotton fiber development. The results confirmed that the expression of some GhTALE genes such as those homologous to *GhKNAT7*, *GhBLH6*, *GhBEL1*, and *GhBLH5* were consistent with formation of FS. Additionally, the genome-wide QTL colocalization of GhTALE genes confirmed the association between GhTALE genes and FS formation from a genetic perspective. Of course, because a 25-cM chromosomal hotspot region may contain several hundred genes [38, 39], the colocalization of a fiber SCW-related trait QTL with a GhTALE gene may not indicate a causal relationship between the natural variation in the TALE genes and FS and/or cell WT. This requires us to select the appropriate populations (including interspecific or intraspecific segregation populations, or even natural populations) in our future research to verify the correlation between the diversity of candidate gene sequences and target traits, which will break the limitation of simple colocalization region screening and provide a genetic basis for further confirmation of functions and possible regulatory molecular mechanisms of target genes. All the above results show the conserved but redundant functions of TALE genes in regulating cotton SCW growth and development.

### The relationship between the cotton fiber SCW and the sclerenchyma SCW

Most of the published research on cotton fiber has focused on fiber initiation and elongation. Little is known about the formation of cotton FS, much less the regulatory network of cotton fiber SCW biosynthesis. Based on the studies of *A. thaliana*, cotton fibers, epidermis hair, trichome initiation and elongation of dicotyledons are well understood, but the cotton fiber SCW contains a high content and purity of cellulose, which is different from the SCW of all *Arabidopsis* cell types; these latter cell types contain a certain proportion of cellulose, hemicellulose, lignin and pectin, meaning that it is difficult to mechanically apply the model plant (*A. thaliana*) model of SCW biosynthesis regulation to understand the regulatory network of biosynthesizing the cotton fiber SCW. Due to the conservation of TALE protein and nucleotide sequences, the TALE proteins should be functionally conserved in identifying downstream DNA sequences even in different species. On the other hand, as lignin has a certain content in the cotton fiber PCW but almost none in the fiber SCW, the inhibitory effect of TALE proteins on lignin synthesis maintains a low-lignin environment to promote the formation of the SCW in cotton fiber. This interpretation reasonably explains the dominant repression of GhKNL1 making fibers shorter and SCWs thinner in previous studies [36].

The article "Genome-wide identification and characterization of TALE superfamily genes in cotton reveals their functions in regulating secondary cell wall biosynthesis" was retracted in 2024. Reasons: duplicated images; original data or images not available; unreliable results or conclusions; concerns about the data.

The published transcriptome data showed that many of the GhTALE genes in upland cotton were expressed at significantly high levels in specific tissues and organs, including class I KNOX KNAT1 subgroup homologs in leaves, class II KNOX KNAT7 subgroup homologs in stems and thickening fibers and the BEL1-like member BLH4 in stems and thickening fibers, suggesting that GhTALE genes may play an important role in leaf, stem and fiber development, similar to their homologs in *A. thaliana* (Fig. 4a). The candidate SCW-related GhTALE genes exhibited varied levels of expression in the thickening period fiber of accessions with differences in FS, which provided proof that GhTALE proteins participate in the regulation of cotton fiber SCW biosynthesis. In summary, the function of TALE proteins may be conserved in different species, but the regulatory mechanisms of cotton SCW biosynthesis often have the species specificity for *Gossypium* and even tissue specificity for cotton fiber cells.

### TALE proteins may simultaneously participate in the regulation of Verticillium wilt resistance and cell wall biosynthesis

Lignin is synthesized by oxidative coupling of three monolignols, p-hydroxyphenyl (H), guaiacyl (G), and syringyl (S) monomers. The proportion of these three main units in the cell wall varies according to plant species and tissue types. Plants enhance cell walls by altering monomer composition and cross-linking, thus adopting effective mechanisms to restrict the spread of pathogens in vascular structures. Xu et al. (2011) identified the central role of lignin metabolism in cotton resistance to *Verticillium dahliae* [59]. In accordance with these reports, it was suggested that increased lignification and cross-linking of resistant cotton stems help them to restrict pathogen growth in the vasculature. As TALE proteins play a significant role in the regulation of lignin biosynthesis, especially in cotton stem vascular tissues, we speculate that the TALE family genes also play a role in the regulation of Verticillium wilt resistance in cotton.

In addition, to determine whether these GhTALE genes are genetically involved in Verticillium wilt resistance in cotton, we also performed a genome-wide colocalization analysis of all GhTALE TFs with Verticillium wilt resistance (VW) QTLs on TM-1 chromosomes. There were 126 and 42 VW QTLs from intraspecific upland populations and interspecific *G. hirsutum* × *G. barbadense* populations, respectively, and they were downloaded for analysis (Additional file 7: Table S4). Interestingly, many VW QTLs clearly share the same regions (QTL clusters) with SCW-related QTLs, and the vascular cell wall structure being associated with pathogen resistance indicates that some genes are bridges or common factors of these regulatory pathways. GhKNAT7-A12 was in a QTL cluster region for both VW and FS QTLs (Fig. 4a-b). As previously reported, GhPFN2, a fiber-preferential actin-binding protein that can interact with the BEL1-like homeodomain protein BLH4, enhanced protection against *Verticillium dahliae* invasion in cotton [60]. Moreover, overexpression of *GhPFN2* promoted the progression of developmental phases in cotton fibers, and the overexpression transgenic lines exhibited stronger secondary wall deposition than the wild type [61]. In addition, the *Arabidopsis* homologs of *GhMYB46*, which is a direct regulator of many TALE family genes, also play a pivotal role in regulating pathogen susceptibility [62]. In conclusion, this information improves our understanding of the regulation of TALE family genes that participate in both Verticillium wilt resistance and SCW biosynthesis.

The article "Genome-wide identification and characterization of TALE superfamily genes in cotton reveals their functions in regulating secondary cell wall biosynthesis" was retracted in 2024. Reasons: duplicated images; original data or images not available; unreliable results or conclusions; concerns about the data.

### The complex interactions of TALE proteins in regulating fiber SCW biosynthesis

In this work, overexpression of *GhKNAT7-A03* and *GhBLH6-A13* (homologs of *AtKNAT7* and *AtBLH6*) in transgenic *Arabidopsis* resulted in a similar phenotype as *A. thaliana* with overexpression of the homologous genes. This result indicated that the functions of TALE genes in cotton might be in line with those in *Arabidopsis*. Moreover, KNAT7 interacts with BLH6 to form a heterodimer that regulates SCW biosynthesis and is functionally conserved in *Arabidopsis* and *Populus* [24]. In addition to the formation of KNOX/BELL complexes between members of the TALE superfamily proteins, KNAT7 can also interact with members of other transcription factor families (such as the MYB or OFP families) to regulate SCW formation. For example, the interacting MYB75 and KNAT7 TFs modulate SCW deposition both in stems and seed coats in *Arabidopsis* [25]. The present study shows that the TALE proteins exhibit some conserved and some different heteromeric interactions in cotton compared with *Arabidopsis*, and some new regulatory mechanisms may be present in the TALE family in cotton. Further studies should be conducted to determine the complete network of interactions.

The article "Genome-wide identification and characterization of TALE superfamily genes in cotton reveals their functions in regulating secondary cell wall biosynthesis" was retracted in 2024. Reasons: duplicated images; original data or images not available; unreliable results or conclusions; concerns about the data.

In the early stages of plant evolution, the BEL1-like and KNOX families proteins have split [63]. In *Arabidopsis*, several AtOFPs interact with members of both TALE families as regulators or cofactors supports the conserved functional connection [64]. A conserved domain at the C-terminal of the AtOFP proteins has been identified to mediate the interaction with the homeodomains of both TALE families proteins [51]. Previously study also showed that the metazoan protein homeodomains involved in both DNA-binding and protein-protein interactions [65]. Evolutionary conservation of BEL1-like and KNOX protein interactions with OFPs to regulate SCW biosynthesis is corroborated in various species; for example, AtOFP1 and AtOFP4 can enhance the repression activity of AtBLH6 by physically interacting with AtBLH6 and AtKNAT7 to form a putative multiprotein transcription regulatory complex regulating SCW formation in *A. thaliana* [66]. In addition, GhKNL1 (also named GhKNAT7-A/D08 in this work), a homeodomain protein in cotton (*G. hirsutum*), is preferentially expressed during SCW biosynthesis in developing fibers, and Y2H assays showed that GhKNL1 can interact with GhOFP4 as well as with its *Arabidopsis* homologs AtOFP4 [36]. In rice, OsOFP2 was expressed in plant vasculature and could interact with putative vascular development KNOX and BEL1-like proteins, so it is likely that OsOFP2 modulates KNOX-BELL function to control diverse aspects of development, including vascular development [67].

In summary, the heteromeric KNAT7-BLH and KNAT7-MYB interactions and the trimeric KNAT7-BLH-OFP interaction have been identified to regulate SCW biosynthesis in different species. The functional conservation of these interaction models will help us explore the complex regulatory network of cotton fiber secondary wall formation more deeply.

### A model for TALE protein involvement in the regulation of cotton growth and development

Fiber strength is a key trait that determines fiber quality in cotton, and it is closely related to SCW biosynthesis. A better understanding of the transcriptional regulatory network of cotton fiber SCW can help us understand the mechanism underlying FS formation. In the present study, combined with previous discoveries, we produced a model network of the TALE family involved in regulating SCW biosynthesis. The findings suggest that GhTALE proteins (including BEL1-like and KNOX proteins) regulate stem sclerenchyma SCW and cotton fiber SCW development by forming heterodimers, and as the core of the regulatory network, GhKNAT7 also interact with OFP1, OFP4 and MYB75 TFs to regulate downstream target lignin and cellulose biosynthesis-related gene expression [36]. GhTALE proteins also act as downstream targets of MYB (GhMYB46) and NAC (GhFSN1) TFs, which were reported to be involved in the regulation of cotton fiber SCW formation (Fig. 8) [37, 62]. Clarification the model of TALE protein actions in combination with progress in cotton genomics may help to elucidate molecular mechanisms for controlling the biosynthesis of cotton fiber SCW and further provide genetic resources for improving cotton fiber quality.

The article "Genome-wide identification and characterization of TALE superfamily genes in cotton reveals their functions in regulating secondary cell wall biosynthesis" was retracted in 2024. Reasons: duplicated images; original data or images not available; unreliable results or conclusions; concerns about the data.

**Fig. 8:** Schematic model of TALE superfamily genes involved in the regulation of cotton growth and development. In plants, TALE proteins always form heterodimers (BEL1-like proteins binding KNOX proteins) to regulate plant growth and development. KNAT7 plays a central role in regulating cotton fiber SCW biosynthesis and can interact with BEL1-like members (including BEL1, BLH1, BLH5, and BLH6) and other TFs (including OFP1, OFP4 and MYB75) to form a complex. Moreover, the TALE heterodimers are often directly targeted by *GhMYB4*6 and *GhFSN1* genes. Downstream of this pathway, TALE heterodimers directly bind the promoters of some lignin and cellulose biosynthesis genes to regulate the thickening of fiber secondary cell walls. The solid lines represent the findings of this study and the dashed lines represent the discoveries of previous studies

## Conclusion

In the present study, a total of 46, 47, 88 and 94 TALE superfamily genes were identified in *G. arboreum*, *G. raimondii*, *G. barbadense* and *G. hirsutum,* respectively. Phylogenetic and evolutionary analysis showed the evolutionary conservation of two cotton TALE families (including BEL1-like and KNOX families). Gene structure analysis also indicated the conservation of GhTALE members during genetic evolution. The analysis of promoter cis-elements and expression patterns suggested potential transcriptional regulation functions in fiber SCW biosynthesis and responses to some phytohormones for GhTALE proteins. Genome-wide analysis of colocalization of TALE transcription factors with SCW-related QTLs revealed that some BEL1-like genes and KNAT7 homologs may participate in the regulation of cotton fiber strength formation. Overexpression of *GhKNAT7-A03* and *GhBLH6-A13* significantly inhibited the synthesis of lignocellulose in interfascicular fibers of *Arabidopsis*. Yeast two-hybrid (Y2H) experiments showed extensive heteromeric interactions between GhKNAT7 homologs and some GhBEL1-like proteins. Yeast one-hybrid (Y1H) experiments identified the upstream GhMYB46 binding sites in the promoter region of GhTALE members and defined the downstream genes that can be directly bound and regulated by GhTALE heterodimers. In summary, this study provides important clues for further elucidating the functions of TALE genes in regulating cotton growth and development, especially in the cotton fiber SCW biosynthesis network, and it also contributes genetic resources to the improvement of cotton fiber quality.

The article "Genome-wide identification and characterization of TALE superfamily genes in cotton reveals their functions in regulating secondary cell wall biosynthesis" was retracted in 2024. Reasons: duplicated images; original data or images not available; unreliable results or conclusions; concerns about the data.

## Methods

### Plant materials and growth conditions

Upland cotton TM-1 was used for gene cloning, a tissue/organ quantitative real-time RT-PCR analysis was used three upland cotton cultivated species (*Gossypium hirsutum* cv. TM-1, Ken 27 and Suyou 6018) which were grown at Anyang (AY), Henan, China, fiber samples were collected at 10, 20 and 30 DPA for RNA extraction. All cotton cultivated species are from and kept in our laboratory.

The transformation of *Arabidopsis thaliana* was carried out by using *Arabidopsis* ecotype Col-0 as the parent. The seeds to be screened were sown in 1/2 Murashige and Skoog (MS) medium after surface disinfection and cultured at 4 °C for 3 days in dark to break dormancy. Then the plants were transferred to a environment with 22 °C, 16-h light/8-h dark photoperiod and about 80% humidity cultured.

### Prediction and cladistic analyses of TALE superclass genes

The genome sequences of *G. raimondii* (D5), *G. arboreum* (A2), *G. hirsutum* acc. TM-1 (AD1) and *G. barbadense* acc. H7124 (AD2) were downloaded from the CottonGen website (https://www.cottongen.org/). To identify potential TALE proteins in the four cotton species, all the TALE amino acid sequences from *Arabidopsis* were used as search queries in local BLAST (with an threshold value of E ≤ 1e-5) searches individually against all four cotton genome databases, and the collected TALE-like candidates were subjected to a further selection based on their conserved domain using SMART (http://smart.embl-heidelberg.de/). MEGA 6.0 (http://www.megasotware.net/) was used to generate minimal evolutionary trees for phylogenetic analysis of TALE superfamily members, and 1000 repetitions of bootstrap analysis were performed. The Ka/Ks ratio was used to assess the selection pressures for duplicate genes and was calculated by the Ka/Ks_Calculator.

### In-silico mapping and analysis of TALE genes

MapChart software (http://www.earthatlas.mapchart.com/) was used to visualize the distribution of the GhTALE genes and QTLs on the *G. hirsutum* chromosomes, A01 to A13 (or c1 to c13) and D01 to D13 (or c14 to c26). In the present study, colocalization of predicted Upland cotton GhTALE genes with QTLs for fiber strength (FS) and wall thickness (WT) were used to screen for potential GhTALE genes that may be involved in fiber SCW development in cotton. QTLs in this paper were downloaded from CottonQTLdb (http://www.cottonqtldb.org), the QTL regions on the sequenced TM-1 genome were confirmed by their flanking marker sequences or primers.

The article "Genome-wide identification and characterization of TALE superfamily genes in cotton reveals their functions in regulating secondary cell wall biosynthesis" was retracted in 2024. Reasons: duplicated images; original data or images not available; unreliable results or conclusions; concerns about the data.

### Gene structure analysis and conserved motif identification

The exon/intron structures of GhTALEs were drawn using GSDS 2.0 (http://gsds.cbi.pku.edu.cn/) through inputting genes GFF files [68]. MEME (Version 5.0.2) (http://meme-suite.org/) was employed to identify conserved motifs of GhTALEs with the following parameters: The maximum number of motifs was 20, and the optimum width was from 6 to 250.

### Analysis of cis-acting elements and TFBSs in the promoter region

TALE genes identified from upland cotton, including their predicted promoter sequences, were downloaded from the CottonGen website (https://www.cottongen.org). The putative cis-acting elements in the promoter regions (1.5 kb upstream from the start codon) were predicted using PlantCARE (http://bioinformatics.psb.ugent.be/webtools/plantcare/html/) software as previously described.

PlantPAN 2.0 database (http://plantpan2.itps.ncku.edu.tw/) was used to identify the putative TFBSs in the predictive promoter sequences (2.0 kb upstream from the start codon) of all GhTALE genes and the structural genes of the lignin and cellulose biosynthesis pathway, and the identified cis-element sequences were manually double-checked against original references; element sequences containing inconsistencies were discarded.

### Expression pattern analysis

To analyze the expression patterns of GhTALE genes, we used RNA-Seq data from *G. hirsutum* acc. TM-1, including data from root, stem, leaf, tours, ovules (− 3, 0 and 3 DPA, days post anthesis) and fibers (5, 10, 20 and 25 DPA). The expression levels of GhTALE genes were calculated using log2 (FPKM).

### RNA isolation and quantitative RT-PCR analysis

Total RNA was extracted from fibers (10, 20 and 30 DPA). RNA was purified using the RNAprep Pure Plant Kit (TIANGEN) according to the manufacturer’s instructions. First-strand synthesis of cDNA was synthesized from 2 μg of total RNA using ReverTra Ace qPCR RT Kit (Toyobo). The qRT-PCR experiments were conducted using 5 fold diluted cDNA template and to measure the expression of related cotton genes in developmental fibers. A cotton polyubiquitin gene (*GhHis3*, GenBank accession no. AF024716) was used as the internal control for the RT-PCR. PCR was performed using SYBR Green Real-Time PCR Master Mix (Toyobo) according to the manufacturer’s instructions, and gene-specific primers used for qRT-PCR analysis are listed in Additional file 10: Table S7.

### Vector construction and plant transformation

To generate transgenic plants overexpressing *GhKNAT7* and *GhBLH6*, the full-length CDSs of *GhKNAT7-A03* and *GhBLH6-A13* were amplified from upland cotton TM-1 cDNA and inserted into the BamHI and SacI restriction sites of the binary vector pBI121, which contains the 35S promoter. The resulting constructs, pBI121:*GhKNAT7-A03* and pBI121:*GhBLH6-A13*, were introduced into the *A. tumefaciens* strain LBA4404. Columbia (Col-0), an *Arabidopsis* ecotype, was transformed using the floral dip method [69]. The transgenic seeds were selected on 1/2 MS medium-containing plates supplemented with 40 mg L^− 1^ kanamycin. The primers used for cloning and vector construction are listed in Additional file 10: Table S7.

The article "Genome-wide identification and characterization of TALE superfamily genes in cotton reveals their functions in regulating secondary cell wall biosynthesis" was retracted in 2024. Reasons: duplicated images; original data or images not available; unreliable results or conclusions; concerns about the data.

### Yeast two-hybrid assay

For directed Y2H assays testing protein-protein interactions between GhKNAT7 proteins and selected GhBEL1-like proteins, due to the high similarity in the amino acid sequences of GhBEL1-like and GhKNOX homologs in the At subgenome and Dt subgenome, we performed PCR-based cloning for any one of the GhTALE homologs, the coding sequences of these proteins were amplified by PCR using GXL DNA polymerase and gene-specific primers (Additional file 10: Table S7) and then cloned into the Y2H vectors pGBKT7 (bait vector) and pGADT7 (prey vector), creating fusions to the binding domain and the activation domain of the yeast transcriptional activator GAL4, respectively. Each BEL1-like/KNOX pair was individually cotransformed into Y2H yeast cells. The transformants were further streaked on quadruple dropout medium (DDO medium, SD/−Trp/−Leu and QDO medium, SD/−Trp/−Leu/−His/−Ade).

### Yeast one-hybrid assay

The Y1H assays were performed as described [70]. Briefly, the ORFs of *GhMYB46-A13* and *GhKNAT7-A03* were each cloned into the pGADT7 vector. Three times of the predicted GhMYB46/GhKNAT7 binding site sequences, e.g., M46-B1 (gtTAGGTt), M46-B2 (cAACCAcc), K7-B1 (gtTGACAgca) and K7-B2 (aTGTCAag), were each constructed into the pHIS2 vector. A constructed pGADT7 prey vector and a corresponding pHIS2 bait vector were cotransformed into Y187 yeast cells. The transformants were further streaked on SD medium (DDO medium, SD/−Trp/−Leu, and TDO medium, SD/−Trp/−Leu/−His with or without 3-amino-1,2,4-triazole (3-AT)) plates.

## Supplementary information

**Additional file 1: Fig. S1.** Phylogenetics, gene structure, motif analysis, promoter cis-elements and expression patterns of GhKNOX genes.

**Additional file 2: Fig. S2.** The predicted cis-elements of GhTALE gene promoters and the expression of selected GhTALE genes in response to phytohormone treatment.

**Additional file 3: Fig. S3.** A genome-wide analysis of colocalization of all GhTALE genes in the sequenced genome TM-1 chromosomes with QTL hotspots for fiber strength (FS) and wall thickness (WT) traits in intraspecific upland cotton populations and interspecific *Gh* × *Gb* populations.

The article "Genome-wide identification and characterization of TALE superfamily genes in cotton reveals their functions in regulating secondary cell wall biosynthesis" was retracted in 2024. Reasons: duplicated images; original data or images not available; unreliable results or conclusions; concerns about the data.

**Additional file 4: Table S1.** *G. hirsutum* TALE superfamily genes and its orthologues in *Gb*, *Ga* and *Gr* cotton genomes.

**Additional file 5: Table S2.** The detailed information of Ka/Ks for TALE family homologs in different *Gossypium* species.

**Additional file 6; Table S3.** The QTLs of FS and WT in intraspecific upland cotton populations and interspecific *Gh* × *Gb* populations.

**Additional file 7: Table S4.** The QTLs of VW in intraspecific upland cotton populations and interspecific *Gh* × *Gb* populations.

**Additional file 8: Table S5.** The cis-element analysis of GhTALE gene promoters.

**Additional file 9: Table S6.** TFBSs analysis of GhKNAT7 and GhMYB46 in the structural gene promoters of the lignin and cellulose biosynthesis pathway and GhTALE family gene promoters.

**Additional file 10: Table S7.** Primer sequences were used in this study.

## Data Availability

All data generated or analysed during this study are included in this published article and its Additional files.

## Abbreviations

aa: amino acid
DPA: days post anthesis
FPKM: fragments kilobase of exon model per million mapped reads
GA: Gibberellic acid
JA: jasmonate acid
Ka: substitution rate of non-synonymous
Ks: substitution rate of synonymous
NJ: neighbor joining
qRT-PCR: quantitative real-time PCR
QTLs: Quantitative trait loci
SA: salicylic acid
SCW: secondary cell wall
TALE: three-amino-acid-loop-extension
TFs: transcription factors
